# Efficacy of Rosuvastatin Combined with rt-PA Intravenous Thrombolytic Therapy for Elderly Acute Ischemic Stroke Patients

**DOI:** 10.1155/2022/9403693

**Published:** 2022-06-15

**Authors:** Jianzhong Zhu, Shan Wang, Zhenqiu Chen, Qiqi Cheng

**Affiliations:** ^1^Department of Neurology, Longmen County People's Hospital, Huizhou 516800, Guangdong Province, China; ^2^Department of Cardiovascular Medicine, Longmen County People's Hospital, Huizhou 516800, Guangdong Province, China

## Abstract

**Background:**

Acute ischemic stroke (AIS) is a fatal and disabling disease. Given the unsatisfactory results by current treatment strategies, optimizing the treatment of AIS is still an urgent problem to be solved.

**Objective:**

To determine the therapeutic efficacy of rosuvastatin (ROS) combined with thrombolytic therapy using recombinant tissue plasminogen activator (rt-PA) on senile AIS patients and analyze its effects on serum inflammatory responses and neurological function.

**Methods:**

A retrospective study was conducted on 150 senile AIS patients who visited the Longmen County People's Hospital between January 2019 and June 2021. Of them, 100 cases treated by ROS combined with rt-PA intravenous thrombolytic therapy (ivTT) were set as the observation group and the rest 50 cases receiving rt-PA alone were included in the control group. Intergroup comparisons were conducted with respect to the following parameters: neurological function (National Institutes of Health Stroke Scale, NIHSS; Scandinavian Stroke Scale, SSS), serum neuron-specific enolase (NSE) and high-sensitivity C-reactive protein (hs-CRP), therapeutic efficacy, incidence of adverse reactions, and patient satisfaction.

**Results:**

The observation group had lower NIHSS and SSS scores and serum NSE and hs-CRP than the control group. In addition, the observation group was found with a higher overall response rate, higher patient satisfaction, and fewer adverse reactions.

**Conclusion:**

ROS combined with rt-PA ivTT can better enhance the therapeutic efficacy of elderly patients with AIS, improve their neurological function, and reduce serum inflammatory responses.

## 1. Introduction

Stroke is a fatal disease that accounts for 5% of disability and 10% of deaths worldwide [1, 2], of which approximately 80% are ischemic strokes [3, 4]. Acute ischemic stroke (AIS) is most prevalent, which can lead to disability due to adverse events such as ischemic injury and neuronal cell death [5]. The risk of this common cardiocerebrovascular disease increases with age [6, 7]. According to epidemiological data, the global incidence of stroke increased by 70-85% from 1990 to 2019, and the number of deaths increased by nearly 45%, with about 795,000 people in the United States being affected by the disease every year [8]. Stroke is attributed to intracranial vascular occlusion induced by atherosclerosis, which prevents blood from flowing into a part of the brain, leading to ischemic necrosis of this part of brain tissue [9, 10].

The prognosis of stroke is poor in middle-aged and elderly patients [11, 12]. Besides, such a disease will not only significantly lower the quality of life of patients but also affect their normal movement function and even consciousness, eventually leading to disability or death [13, 14]. Therefore, the treatment of stroke has always been an important direction of clinical research.

Clinically, statins are commonly used to treat cardiovascular diseases because of their cholesterol-lowering effect on blood vessels, as well as antiangina pectoris and anti-ischemic properties [15]. They can inhibit the formation of mevalonate pathway and isoprenoid, prevent endothelial ischemia-reperfusion injury, improve endothelial function, enhance ischemic vasodilation, and relieve inflammation [16]. Among them, rosuvastatin (ROS) has an obvious inhibitory effect on inflammatory factors [17]. Recombinant tissue plasminogen activator (Alteplase) (rt-PA), another commonly used drug in cardiocerebrovascular diseases, is a serine protease that can cleave plasminogen to activate plasmin. Although it plays an important role in cardiovascular diseases, its toxicity is prone to cause a series of complications and even ischemia-reperfusion injury after revascularization [18]. Yang et al. [19] reported that ROS combined with rt-PA for patients with AIS, no matter high or low dose of ROS, had no significant effect on their functional outcomes at 3 months, and the safety was comparable. However, the comparative analysis of ROS combined with rt-PA and rt-PA alone in the treatment of AIS is still limited.

Given that there are few related studies on the combination of these two drugs in treating ischemic stroke, we analyzed the effectiveness of the combination therapy for elderly AIS patients. In addition, the novelty of this research lies in the comprehensive comparison and evaluation of the effectiveness and reliability of the combination of the two drugs in the treatment of AIS from the aspects of neurological function, inflammation-related serum indexes, clinical efficacy, safety, and treatment satisfaction, which provides a reliable theoretical reference for AIS treatment.

## 2. Methods

### 2.1. General Information

This retrospective study selected 150 elderly AIS patients who visited the Longmen County People's Hospital between January 2019 and June 2021 and assigned them to observation (*n* = 100) and control (*n* = 50) groups. The general data of the two cohorts were balanced and comparable (*P* > 0.05). The Ethics Committee at the Longmen County People's Hospital approved this research, and patients and their families agreed and signed the informed consent.

Inclusion criteria are as follows: ① diagnosis of AIS in our hospital; ② age > 60; ③ single lesion; ④ first episode, with onset-to-thrombolysis time less than 4.5 h; and ⑤ duration of symptoms and signs of brain dysfunction > 1 h. Exclusion criteria are as follows: ① presence of intracranial hemorrhage as indicated by CT examination; ② history of stroke and major head trauma within the last 3 months; ③ tendency of active bleeding focus or bleeding; ④ intracranial tumors, aneurysms, and arteriovenous malformations; ⑤ recent use of systematic anticoagulant, thrombolytic, and fibrinolytic treatments; ⑥ organic diseases of liver, kidney, heart, and other organs; and ⑦ mental system, immune system, and blood system diseases.

### 2.2. Methods

Before treatment, all patients were given routine treatment, including reducing blood sugar, lowering blood pressure, anti-infection, nourishing nerves, and correcting acid-base and water-electrolyte disorders. Based on that, the control group received intravenous thrombolytic therapy (ivTT) with rt-PA (Boehringer Ingelheim International GmbH, Germany, Import Drug Registration Certificate Nos.: S20110051 and S20110052), with a total dose of 0.9 mg/kg and a maximum of ≤90 mg; 10% of the drug was administered as a single iv bolus within 1 min, and the remaining 90% was given by continuous iv drip within 1 h. The observation group was given ROS (Simcere Pharmaceutical Group Limited, Nanjing, China, SFDA Approval No.: H20113246) in addition to rt-PA ivTT and routine treatment. The thrombolytic therapy was given with the same method and dosage as mentioned in the control group, and in addition to that, oral administration of ROS was given 15 mg/time, once a day for one month after ivTT.

### 2.3. Outcome Measures

#### 2.3.1. National Institutes of Health Stroke Scale (NIHSS) and Scandinavian Stroke Scale (SSS) Scores

The neurological recovery and limb function of patients were analyzed and compared at admission and one month posttreatment. The NIHSS [20] and SSS [21] were used to evaluate patients' neurological function recovery, with lower scores indicating better recovery.

#### 2.3.2. Serum Factors Neuron-Specific Enolase (NSE) and High-Sensitivity C-Reactive Protein (hs-CRP)

The measurement of serum NSE and hs-CRP was conducted upon admission and 7 days after treatment, using human NSE enzyme-linked immunosorbent assay (ELISA) kit and human hs-CRP ELISA kit (Shanghai Yuanmu Biotechnology Co., Ltd., YM-SZ0162, YM-SZ0895), respectively. All related operations were completed by the hospital's professional testing personnel following the instrument and kit instructions.

#### 2.3.3. Curative Effect

The efficacy of patients was evaluated one month after treatment as follows: ineffective: an increase in NIHSS score or a decrease < 18%; effective: decreased NIHSS score by 18%-45% compared with the pretreatment score; markedly effective: decreased NIHSS score by 46%-90% with disability grades 1-3; and clinically cured: a decrease of NIHSS by 91%-100%, with disability grade 0.

#### 2.3.4. Adverse Reactions (ARs)

The ARs occurred during treatment, such as gastrointestinal dysfunction, urinary incontinence, mild elevation of alanine aminotransferase, and poststroke dementia, were counted and compared.

#### 2.3.5. Treatment Satisfaction

Patients' satisfaction testing used a self-made treatment satisfaction questionnaire (total: 100 points), and satisfaction scores were compared. The test content and evaluation criteria were self-made. Evaluation criteria are as follows: 85-100: satisfied, 70-85: basically satisfied, and <70: dissatisfied.

### 2.4. Statistical Methods

Data were statistically processed by SPSS19.0 (Asia Analytics Formerly SPSS China), and differences with *P* < 0.05 were deemed significant. Count data were tested by *χ*^2^. The intergroup comparison of quantitative data denoted by *X* ± *S* was made by the *t* test, and the intragroup comparison before and after treatment was carried out using the paired *t* test. GraphPad Prism 8 (GraphPad Software, San Diego, USA) was used for image rendering.

## 3. Results

### 3.1. General Information

The intergroup comparison showed no obvious differences in a series of general information such as gender, age, BMI, smoking, and drinking (*P* > 0.05) Table 1.

### 3.2. NIHSS and SSS Scores

After investigation, it was found that the NIHSS and SSS scores changed significantly in both groups after treatment, and these scores were lower in the observation group as compared to the control group (*P* < 0.05) Figure 1.

### 3.3. Serum NSE and hs-CRP Levels

The detection of serum NSE and hs-CRP levels revealed that the two indexes had significant changes in both groups after treatment. After treatment, the two indexes decreased statistically in the two groups (*P* < 0.05) and were lower in the observation group (*P* < 0.05) Figure 2.

### 3.4. Efficacy

The comparison of posttreatment efficacy revealed a higher total effective rate in the observation group when compared to the control group (*P* < 0.05) Table 2.

### 3.5. Incidence of ARs

The comparison of ARs revealed a significantly lower incidence of ARs in the observation group compared with the control group (*P* < 0.05) Table 3.

### 3.6. Treatment Satisfaction

The intergroup comparison of treatment satisfaction showed higher patient satisfaction in the observation group as compared to the control group (*P* < 0.05) Table 4.

## 4. Discussion

The choice regarding the treatment of AIS, a disease with high mortality, is undoubtedly essential [22]. It is wise to use thrombolytic drugs to treat such a cardiocerebrovascular disease [23]. In this section, we will analyze the effects of ROS combined with rt-PA ivTT on elderly patients with AIS based on the results obtained here and related literature.

First, the overall efficacy was statistically higher in the observation group when compared to the control group. Al-Kuraishy et al. [24] pointed out in their study that the application of ROS in AIS patients has certain efficacy, which can improve the cardiac metabolism of patients and lower the risk of stroke recurrence. Lu et al. [25] also confirmed the effectiveness of ROS in AIS in animal experiments, mainly reflected in the prevention of blood-brain barrier damage. In addition, obviously improved neurological function was found in both groups after treatment, with lower NIHSS and SSS scores in the observation group. It suggests that the observation group achieved better outcomes due to better neurological recovery. Similarly, M. Safakheil and H. Safakheil [26] reported that ROS has a protective effect on the neurological function of AIS model rats, and this protective mechanism is related to the reversal of oxidative stress imbalance in the body. Cerebral infarction will cause ischemic injury of the brain, followed by vasoconstriction and blood flow reduction induced by inflammatory factors, resulting in endothelial cell injury in the brain area, which will greatly damage the nerve function [27]. Therefore, neurological function is closely associated with the severity and treatment effect of stroke. The rt-PA used in this study is a common rapid thrombolytic therapy, which can achieve the effect of thrombolysis by catalysing profibrinolysin into active fibrinolytic enzyme. However, if this operation is not completed in a short period of time, it will not only lead to poor effects but also bring a series of adverse symptoms [28]. Relevant research on coronary heart disease has found that ROS, with a potent inhibitory effect on related pathways, also has a good effect on vascular endothelial relaxation [29]. Therefore, in this study, the observation group was first given rt-PA for thrombolytic therapy, and then, ROS was applied for vascular endothelial relaxation, which may explain the better recovery of brain endothelial cell damage and higher treatment efficacy in the observation group.

From the perspective of serum-related factors, this study found that although serum hs-CRP was improved to varying degrees in both groups, the improvement was better in the observation group. Previous studies have confirmed that ROS can significantly reduce neuroinflammation after rt-PA treatment in the AIS mouse model and play a protective role in neurological function by exerting anti-inflammatory effects [30]. The role of statins is to inhibit the Rho/ROCK pathway by inhibiting the formation of isoprenoid intermediates, thus increasing the synthesis of endothelial NO, reducing the contraction and proliferation of vascular smooth muscle cells to reduce the formation of thrombosis, and inhibiting a series of cytokines such as inflammatory factors [31]. hs-CRP, an important marker of the body's inflammatory response, is an acute phase protein synthesized by liver cells in the early stage of inflammation. Due to the damage of DE1 vascular endothelial cells in acute cerebral infarction patients, hs-CRP concentration will be significantly increased [32]. Besides, a study on encephalitis found that the level of NSE was closely related to inflammation, and increased levels were associated with more severe inflammation [33]. Combined with our findings, the additional use of ROS may explain better alleviation of inflammatory responses in the observation group.

This study still has some shortcomings. Although patient satisfaction was investigated in this research, we were unable to investigate patients' quality of life and the improvement of specific limb function and psychological anxiety level after treatment due to time constraints. In addition, this is a single-center small sample study, which may have some impact on the accuracy and universality of the reported results. Finally, there is no analysis regarding the long-term follow-up of patients, which if supplemented, will help further understand the impact of the two regimens on the long-term outcomes of these patients. In future research, we will supplement other indicators to improve the research and evaluate patients' quality of life after treatment, so as to optimize the therapeutic scheme to find a new and effective treatment for AIS in the elderly.

## 5. Conclusion

To sum up, ROS combined with rt-PA ivTT contributes to higher curative effects in senile AIS patients, improves neurological function, and reduces serum inflammatory responses.

## Figures and Tables

**Figure 1:** Neurological function of patients: (a) NIHSS score: the posttreatment NIHSS score of the two groups changed significantly and was lower in the observation group compared with the control group (*P* < 0.05). (b) SSS score: a statistical decrease in SSS score was observed in both groups after treatment, with a lower one in the observation group (*P* < 0.05). Note: ∗ denotes *P* < 0.05 vs. the control group; # denotes *P* < 0.05 vs. after treatment within the group.

**Figure 2:** Serum NSE and hs-CRP levels in two groups: (a) NSE was significantly lower in the observation group than in the control group (*P* < 0.05). (b) Lower hs-CRP was found in the observation group compared with the control group (*P* < 0.05). Note: ∗ denotes *P* < 0.05 vs. the control group; # denotes *P* < 0.05 vs. after treatment within the group.

**Table 1:** General information.

Classification	Observation group (*n* = 100)	Control group (*n* = 50)	*t*/*χ*^2^	*P*
Gender			0.14	0.710
Male	69 (69.00)	33 (66.00)		
Female	31 (31.00)	17 (34.00)		
Age (years)	68.65 ± 3.48	68.28 ± 3.89	0.59	0.556
BMI (kg/m^2^)	23.69 ± 3.42	23.37 ± 3.65	0.53	0.598
Residence			0.06	0.807
Urban	66 (66.00)	34 (68.00)		
Rural	34 (34.00)	16 (32.00)		
Drinking			0.02	0.897
Yes	73 (73.00)	36 (72.00)		
No	27 (27.00)	14 (28.00)		
Smoking				
Yes	69 (69.00)	33 (66.00)	014	0.710
No	31 (31.00)	17 (34.00)		

**Table 2:** Total effective rate after treatment.

	Observation group (*n* = 100)	Control group (*n* = 50)	*χ* ^2^	*P*
Clinically cured	67 (67.00)	21 (42.00)	-	-
Markedly effective	17 (17.00)	12 (24.00)	-	-
Effective	13 (13.00)	8 (16.00)		
Ineffective	3 (3.00)	9 (18.00)	-	-
Total effective rate	97 (97.00)	41 (82.00)	10.19	0.001

**Table 3:** Incidence of adverse reactions after treatment.

	Observation group (*n* = 100)	Control group (*n* = 50)	*χ* ^2^	*P*
Gastrointestinal dysfunction	1 (1.00)	2 (4.00)	-	-
Urinary incontinence	0 (0.00)	3 (6.00)	-	-
Mild elevation of alanine aminotransferase	0 (0.00)	2 (4.00)	-	-
Poststroke dementia	3 (3.00)	4 (8.00)		
Incidence of adverse reactions	4 (4.00)	11 (22.00)	12.00	<0.001

**Table 4:** Patient satisfaction.

Classification	Observation group (*n* = 100)	Control group (*n* = 50)	*χ* ^2^	*P*
Satisfied	70 (70.00)	23 (46.00)	-	-
Basically satisfied	25 (25.00)	16 (32.00)	-	-
Dissatisfied	5 (5.00)	11 (22.00)	-	-
Satisfaction (%)	95 (95.00)	39 (78.00)	10.11	0.002

## Data Availability

The simulation experiment data used to support the findings of this study are available from the corresponding author upon request.
